# An approach toward public hospital performance assessment

**DOI:** 10.1097/MD.0000000000004688

**Published:** 2016-09-09

**Authors:** Vitalis Chukwudi Nwagbara, Rajah Rasiah, Md. Mia Aslam

**Affiliations:** a Institute of Graduate Studies; b Department of Development Studies; c Department of Economics, University of Malaya, Kuala Lumpur, Malaysia.

**Keywords:** health care policy, Malaysia, performance, public hospitals, utilization

## Abstract

**Background:**

Public hospitals have come under heavy scrutiny across the world owing to rising expenditures. However, much of the focus has been on cutting down costs to raise efficiency levels. Although not denying the importance of efficiency measures, this article targets a performance issue that is relevant to address the quality of services rendered in public hospitals. Thus, it is important to focus on the effectiveness of resource utilization in these hospitals. Consequently, this article seeks to examine the impact of average length of stay (ALOS) and bed turnover rates (BTR) on bed occupancy rates (BOR).

**Methods:**

Public hospital inpatient utilization records during the period 2006 to 2013 were gathered from the Ministry of Health, Malaysia. A 2-step generalized method of moments (GMM) statistical method was used to analyze the data. BOR was adopted as the dependent variable, whereas BTR and ALOS were used as the explanatory variables. The logarithm of total bed count (BED), admission (ADM), and patient days (PD) was deployed as control variables. Three regression models were developed to explore the correlates of BOR as a hospital performance measure. Ethics committee approval was waived because no patients were identified in the study.

**Results:**

The statistical analyses show that ALOS and BTR are inversely correlated with BOR, with both coefficients significant at 1%. The control variables of BED, ADM, and PD had the right positive signs and they were significant in both sets of equations. Hence, reducing ALOS and BTR can help raise performance of public hospitals in Malaysia.

**Conclusion:**

In light of the robust results obtained, this study offers implications for improving public hospital performance. It shows a need to reduce ALOS and BTR in public hospitals to improve BOR.

## 1 Introduction

Public hospital management has been an insufficiently explored area of study despite its importance in meeting the health care needs of society. Although organizational behavior theory^[1]^ posits that the internal attributes of organizations should form the basis for performance assessment, it has not been fully applied to the public health care system. Public hospitals serve as a major conduit in the delivery of medical services, as well as account for the largest share of total health care expenditure of countries.^[2]^ Given rising expectations of patients and other stakeholders, the need for improvement in health care delivery has become paramount, especially in the effective use of resources.^[3]^ However, scholars have been divided on the best approaches to assess health care performance,^[1,4]^ which consequently has led to the advocacy of different health care management strategies.^[5]^

The most widely applied approaches are built around the concept of efficiency. This concept originated from the “economic good” theoretical viewpoint.^[6]^ Under this approach, health care is defined mainly by dollars and cents to protect stakeholders’ interests. Hence, financial measures are used as indicators of performance. The underlying estimation method has been to model the maximum attainable outcome through a production function, and to consider any distance from the production possibility frontier as a measure of inefficiency.^[2,7]^ Although being efficient is good for any organization, conventional efficiency measures are not bereft of shortcomings,^[8]^ especially when applied to public hospitals. Given that public hospitals exist mainly to service the health care needs of society,^[2,7]^ their assessment therefore should be tied to their objectives.

However, identifying the appropriate performance measures for public health care organizations, especially public hospitals, has been a challenging task for researchers. Nevertheless, a safe way of addressing the problem is to look inward and focus on the internal dimensions underpinning organizational behavior rather than to simply use the traditional efficiency concepts used in economics. Thus, several studies have relied on bed occupancy rate (BOR) as a major indicator of hospital performance.^[9,10]^ BOR represents the percentage of installed beds occupied in hospitals within a given year, which is used as an indicator of utilization and productivity. The influence of BOR on hospital outcomes has been reported in a number of studies.^[11–13]^

Efforts have been made in the past to model the relationship between hospital service demand and available capacity.^[14]^ Studies in this line of thought suggested risks inherent in a hospital's inability to provide sufficient number of beds to patients. This will then result in BOR overshooting, which will generate negative impacts.^[10,11,15,16]^ An innovative study by Bagust et al^[14]^ established that when BOR exceeds the safe level of 85%, it results in increased chances of access block, long waiting times, and high mortality. BOR above the threshold of 85% would generate overstretched quality of hospital care. This will produce negative consequences, which does not bode well for public hospitals. However, a BOR of <80% is considered to be low and it indicates idleness of facilities.

From the foregoing arguments, the application of BOR as a measure of hospital performance^[9]^ is appropriate. However, its correlates with the average length of stay (ALOS) and bed turnover rates (BTR) have not been statistically proven. Therefore, this article attempts to contribute to the literature on the use of BOR as a hospital performance measure. Because BOR is not a stand-alone measure, understanding its correlates with ALOS and BTR is necessary to contextualize it as a public hospital performance measure. Thus, the overarching goal of this study is to produce estimates that better reflect true, underlying BOR effects as a measure of public hospital performance. This study is relevant because apart from filling the gap in knowledge, it will help policy-makers in hospital capacity planning and utilization.

## 2 Methods

### 2.1 Source of data

The data used in this study were obtained from the Ministry of Health (MOH), Malaysia, and consist of all public hospitals in Peninsular Malaysia during the period 2006 to 2013. Peninsular Malaysia consists of 11 out of the 13 states that make up the country. Public teaching hospitals, public military hospitals, public clinics, private hospitals, polyclinics, and other private health care providers are excluded because the objective is to assess the performance of public hospitals under MOH. It is believed that stronger conclusions on public hospital performance would warrant widening the study period instead of simply carrying out a cross-sectional assessment undertaken by many previous studies. Hence, the article uses longitudinal data and follows panel data analysis model.

### 2.2 Specification of variables

The analysis considers the following variables: BOR, ALOS, BTR, number of beds (BED), admission (ADM), and patient days (PD). It is believed that these constitute a reasonable set of performance measures tailored to public hospitals’ goals of providing care to all and serve as macrolevel hospital performance measures.^[17]^ BOR is adopted as the dependent variable, whereas ALOS, BTR, BED, ADM, and PD serve as independent variables as in earlier studies.^[18,19]^ These measures, which span across utilization, productivity, and quality, serve as proxy indicators of performance and qualify as performance assessment measures.^[1]^ They are hospital-wide measures that denote the general performance of hospitals rather than specific areas of clinical concern. Furthermore, these variables seek to offer insights into some aspects of wastefulness in the use of resources.^[20]^

1. BOR represents the percentage of all licensed and installed beds within a given year, and it is used as an indicator of utilization and productivity. Because performance assessment is a continuous process in any organization, the effects of the previous performance status on the current cannot be discountenanced. Hence, in the ensuing analysis, the first-order lagged term of the BOR (BOR_t−1_) of the dependent variable was presented to control the lagged effect and limit its estimation bias as in Fan et al.^[21]^
2. ALOS has been widely used as an indicator of quality of services provided by hospitals.^[22–25]^ Past studies demonstrate that ALOS is related to cost, efficiency, quality of care, and speed.^[26,27]^ Hence, it is considered as a critical measure of performance. Although neither too long nor too short is desirable, lower values reflect better performance.^[28–30]^ Therefore, ALOS is considered as an indicator driving the BOR. It is measured by dividing the total number of inpatient hospital days by the total number of discharges (including deaths) in all hospitals during a given year. A lower value means a better quality of service, which is helpful in making more beds available to incoming patients. Evidence suggests that significantly lower levels of ALOS and greater number of admissions indicate sound management.^[31]^ This implies that higher BOR which results from higher admissions will have negative correlation with ALOS. Hence, its coefficient is expected to be negative.
3. BTR denotes the number of times each hospital bed changed occupants. It indicates the use made of available hospital beds and has been defined as a measure of productivity.^[32]^ A lower rate may be due to high ALOS; however, when both are very low, it might imply either underutilization or overcapacity. BTR is measured by dividing the total discharges (including deaths) by the total number beds. Because it seems to be of less effect on the dependent variable, its coefficient is expected to be negative.
4. BED includes all installed hospital beds which are regularly maintained, equipped, and staffed, and readily available for the care of admitted patients. Emergency stretchers/bed and beds designated for same-day outpatient care are excluded. This study encompasses different types of public hospitals with varying capacities defined by the number of beds. These variations result in skewness. To limit the effect of the skewness, logarithm (log) of bed is applied. The coefficient associated with bed variable is expected to be positive and statistically significant given that higher capacity will lead to higher admission and utilization and consequently high BOR.
5. ADM refers to *patients* accepted for inpatient services in any of the public hospitals within the period under consideration. As mentioned above, because capacity differs, admissions as well differ and there is skewness in the number recorded in different hospitals. As admission depends on the number of beds which have been found to be skewed, log of ADM is applied.
6. PD refers to units of measure denoting accommodating facilities provided and services rendered to inpatients within the census-taking period. It reflects the volume of services provided by each hospital within a given year. PD impacts the BOR by changing both output and input amounts. So, under the same conditions, higher PD would mean higher utilization and higher BOR. It is assumed that because admission has a potential utilization of hospital resources, increasing PD may generate a larger increasing effect of BOR, and thus can increase the rate of utilization. For these reasons, PD is considered an important factor of BOR. It is calculated as ADM multiplied by ALOS. Its coefficient is expected to be positive.

BED is used as a proxy to capture hospital size effect on BOR. Large-sized hospitals are defined as those having high number of beds. Although ADM depends on other factors, such as location, specialty, and the like, it does represent the quality of the services provided. Better quality of services attracts patients from far and near, and hence could influence BOR. On the contrary, hospitals with reports of poor quality of services will have lesser number of patients in comparison with those providing better quality. Similarly, PD captures the number of days in totality that patients stay in hospitals as inpatients within a given time period. Table 1 shows the descriptive statistics of all the considered variables.

**Table 1:** Descriptive statistics.

The maximum BOR was 132.8%, the minimum was 14.7%, while the mean was 58.0% (Table 1). ALOS on the average had 1.84 and 18.74 days as its minimum and maximum, whereas the mean was 3.26 days. Similarly, BTR recorded a minimum of 12.8 and maximum of 150.4 times with a corresponding mean of 67.20 times. Hospital capacity defined by the number of beds has a minimum and maximum of 20 and 2408, respectively, with a mean of approximately 298.5 implying that on the average, public hospitals in Malaysia range from medium to large sizes. Admission follows the same trend with a minimum of 1286 and maximum of 124,627, whereas the mean was 19,285. Correspondingly, the minimum and maximum PD were 7300 and 878,920 with a mean of 109,459 days.

Table 2 shows evidence of multicollinearity between some of the independent variables, which is an issue associated with panel data models.^[33]^ To overcome the multicollinearity among the explanatory variables of ALOS and BTR, and among the control variables of BED, ADM, and PD and their possible effects, they are separately introduced in the generalized method of moments (GMM) estimation. Hence, to investigate the determinants of BOR, the following static panel data model is considered:      

**Table 2:** Pairwise correlation.

### 2.3 GMM estimation

This article deploys a partial adjustment model to bring the econometric analysis close to practicality. However, the lagged dependent variable (LDV) can lead to endogenous problems because of the correlation between independent variables and the error term. Hence, fixed and random effects are not adopted in order not to bias the results of the panel data estimation. Rather, the GMM estimator, which takes the LDV and past values of other potentially endogenous variables in the regression as instruments, was adopted.^[34]^

Generally, GMM estimation takes account of heteroskadesticity and serial correlation between exogenous variables and error terms.^[35]^ In this study, LDV and endogenous variables are used to form GMM-type instruments. LDV is applied purposely to provide robust estimates of the effects of independent variables and yield more accurate parameter estimates.^[36]^ Adding LDV to a regression model has been demonstrated as a veritable way of helping purge error autocorrelation.^[37]^

Furthermore, considering that the endogenous problem is crucial for the robustness of the estimated results, the system GMM is deployed to ensure that the instruments and moment conditions are rational. It assumes that if the instruments are well selected, there is a first-order serial correlation in the error term, but no second-order correlation.^[21]^ The Arellano–Bond (AB) test is applied to judge the validity of the instruments.

In the diagnostic tests, the Hansen test of overidentification which examines the appropriateness of the instruments used is employed. Similarly, the Arellano–Bond AR (2) test was applied to test the existence of the first- and second-order serial correlation in the first-difference residuals. First differences of the exogenous variables are used as standard instruments as in Roodman.^[38]^ The endogeneity test of the endogenous regressor supports the preference for a 2-stage GMM as applied.^[39]^ Ethics committee approval was waived because no patients were involved in the study.

## 3 Results

To observe the influence of the independent variables on BOR and increase the robustness of the empirical results, the independent variables were introduced into the regressions as shown in models (i) to (vi) above following the practice as used by Fan et al.^[21]^ The results are shown in Tables 3 and 4.

**Table 3:** Relationship between ALOS and BOR, public hospitals, Malaysia, 2006 to 2013.

**Table 4:** Relationship between BTR and BOR, public hospitals, Malaysia, 2006 to 2013.

### 3.1 Findings

In models (i) to (iii), we examine the impacts of the lagged BOR and ALOS in all 3 of them, and the control variables of log of BED, log of ADM, and log of PD separately in each of them to avoid collinearity problems. The Arellano–Bond test indicates that the error terms in all regressions are significant at the first-order, and are serially correlated at the 1% level, but not at the second-order level. Therefore, the above assumption of the system GMM is satisfied. The Hansen test shows that there is no overidentification problem of instrumental variables in all regressions. This implies that the instrumental variables are valid and effective, and thus the estimated results are credible. All coefficients in the 6 models are statistically significant. Thus, the empirical analysis is robust, and the selected determinants are pivotal to BOR.^[21]^

### 3.2 Discussion

As models (i) to (iii) show, the coefficients of ALOS variable (which vary between −0.01 and −0.03), are negative and statistically significant (1%), which confirms our first hypothesis. This implies that an increase in ALOS will not necessarily lead to an increase in BOR, ceteris paribus. Another possible explanation is that keeping patients longer than clinically necessary to increase BOR may not result in better overall public hospital performance. When ALOS is high, it could mean that patients stay longer in hospitals and the same bed cannot be occupied by fresh patients until they are discharged. Furthermore, the evidence shows that lower ALOS enhances BOR performance. In line with previous studies,^[39]^ this finding indicates that a reduction in ALOS improves hospital performance. Although thresholds of ALOS vary with different kinds of treatments, it will require a new study to address such variations as the data used here is aggregated at the hospital level.

As models (iv) to (vi) show, the coefficients of BTR variable (which vary between −0.001 and −0.002) are negative and statistically significant (5%), which confirms our second hypothesis. This implies that an increase in BTR will lower BOR, ceteris paribus. These results show that the raising of BTR, especially involving uncritical treatments, may not lower ALOS (especially when involving critical treatments) as both variables are inversely correlated with BOR.

Hence, ALOS and BTR can both be raised in Malaysian public hospitals to lower BOR. The evidence shows that higher ALOS and BTR enhance BOR performance. A certain threshold of ALOS and BTR may be necessary to establish the optimal BOR of hospital performance. However, such estimations can only be done for the same kind of treatments, which will require a new study as the data used here are aggregated at the hospital level as mentioned above. Such a study would require more direct fieldwork on hospitals, so that a control variable by type of treatment and degree of health danger can be introduced as a control variable.

## 4 Conclusions and implications

Based on the panel data of public hospitals in Malaysia during the period 2006 to 2013, and the GMM regressions, this article estimated the influence of ALOS and BTR on BOR as a hospital performance measure. The results show that there is an inverse relationship between ALOS and BOR on the one hand and between BTR and BOR on the other hand. The results are highly significant after controlling for BED, ADM, and PD. Unlike some previous studies that simply presented the 3 measures of performance separately without a statistical link between them, that is BOR, ALOS, and BTR,^[29,39]^ this exercise went further to analyze the statistical impact of ALOS and BTR, on BOR controlling for BED, ADM, and PD.

The results call for a better understanding of the performance of public hospitals, so that its properties as a social good (public good) can reach everyone.^[40]^ Both ALOS and BTR influence BOR strongly. That ALOS and BTR can be raised to lower BOR suggests that the measurement of efficiency in public hospitals must address effectiveness rather than simply relying on only financial measures related to costs and profits, which should be used when dealing with profit-oriented organizations. During the study period of 2006 to 2013, a maximum of 132.8% and minimum of 14.7% BOR were recorded, which indicates that both overcapacity and undercapacity have characterized public hospitals in Malaysia. This implies poor planning, which calls for better management of the public hospitals in Malaysia.

Another major implication that could be drawn is that the strong inverse relationship between BTR and BOR obtained in this study is also consistent with another finding on private hospitals.^[41]^ However, while the results on ALOS was significant and the coefficient negative in our study of public hospitals, a positive and significant coefficient of ALOS was reported on private hospitals.^[41]^ Thus, it is clear that the management of ALOS in public hospitals may have to address them as created to a social objective without having to comprise on hospital performance (BOR).

The evidence provided in this study suggests that targeted efforts at increasing utilization rates of public hospitals can increase their overall performance, which is in sync with a previous study that showed that reducing hospitalization rates leads to an improvement in efficiency.^[41]^ Therefore, health care policy-makers should ensure a coordinated action plan toward the promotion of health care facility utilization to enhance overall health care delivery.

Following the robust findings, this study proposes some policy measures to improve BOR as an indicator of performance in public hospitals. First, efforts must be taken at increasing the utilization of and improvement of coordination of inpatient admissions at public hospitals. Because the allotment of resources, especially the distribution of hospitals, is highly skewed as evident from differences in the capacity and admission by hospital categories, prudent allocation of resources should be followed by governments and other relevant stakeholders. Second, it is advisable to stimulate the utilization of public hospital facilities carefully as raising ALOS in this study shows improvements in BOR. Thus, health care policy-makers should formulate policies targeted at increasing access to care.

Like any epistemological assessment this study has limitations. Future research is necessary, so that the results are controlled for best practice hospitalization periods on the basis of degree of criticalness (severity) among the patients admitted. Also, future studies should examine the extent to which public hospital performance is influenced by BTR, and how it mediates the relationship between ALOS and BOR.

## Acknowledgments

Our appreciation goes to Dr. Ali Boerhonnoeddin for his unrelenting advice, to University of Malaya for providing the platform to carry out this study. Finally, we wish to thank officials of the Ministry of Health for assisting us in getting the necessary data that helped shape this study.
